The article "Urinary Bladder Hernia: A Rare Cause of Urinary Frequency" was retracted in 2024. Reasons: false authorship; unreliable results or conclusions; no approval from an author; concerns about the authorship.

# Urinary Bladder Hernia: A Rare Cause of Urinary Frequency

**DOI:** 10.7759/cureus.20993

**Published:** 2022-01-06

**Authors:** Abdurahman A Aldubaikhi, Sultan A Albeabe, Ahlam M Alfaraj, Talal M Al Thobaiti, Salman S Shaaban, Thamer S Aloqaili, Alhanouf S Aldossary, Sami N Alanazi, Ziyad F Althobaiti, Ebtehal Z Alqahtani, Abdulrahman Z Alqahtani, Ali S Alsoghayer, Abdulhalim A Alabdullatif, Abdulwahab A Altammar, Faisal Al-Hawaj

**Affiliations:** 1 College of Medicine, Qassim University, Qassim, SAU; 2 College of Medicine, Arabian Gulf University, Manama, BHR; 3 College of Medicine, Jordan University of Science and Technology, Irbid, JOR; 4 College of Medicine, King Abdulaziz University, Jeddah, SAU; 5 College of Medicine, University of Dammam, Dammam, SAU; 6 College of Medicine, AlMaarefa University, Ad Diriyah, SAU; 7 College of Medicine, Northern Border University, Arar, SAU; 8 College of Medicine, Taif University, Taif, SAU; 9 College of Medicine, Jazan University, Jazan, SAU; 10 College of Pharmacy, Jazan University, Jazan, SAU; 11 College of Medicine, University of Malta, Msida, MLT; 12 College of Medicine, Imam Abdulrahman Bin Faisal University, Dammam, SAU

**Keywords:** case report, laparoscopy, bladder hernia, urinary frequency, inguinal hernia

## Abstract

Hernia repair is one of the most commonly performed surgical operations worldwide. Inguinal hernia is a common condition and has a high prevalence rate. Advanced age and male sex are the most important risk factors. Inguinal hernia usually presents with groin swelling with abdominal discomfort. We report the case of a 39-year-old man who presented to our urologic clinic with a complaint of urinary frequency for the last two months. This was associated with nocturia, feeling of incomplete emptying, and groin swelling. There was no history of hesitancy, intermittency, or weak stream. The patient was otherwise healthy with no significant previous medical or surgical history. Abdominal examination showed a right groin swelling with associated visible and palpable cough impulse in keeping with inguinal hernia. There was no abdominal guarding or rigidity, and the abdomen was non-tender. Examination of the genitalia was unremarkable. No abnormal findings were noted in the examination of other systems. Routine laboratory markers did not show any abnormalities. Urinalysis findings showed no leukocytes and had negative results for leukocyte esterase and nitrites. A computed tomography (CT) scan confirmed the presence of a right-sided inguinal hernia, with part of the urinary bladder seen herniating into the right inguinal canal. The patient underwent a laparoscopic surgery in which the herniated bladder was reduced and the defect was closed with a synthetic mesh. The patient recovered with no complications. Postoperatively, the patient reported significant improvement in his symptoms. Herniation of the bladder through the inguinal canal is an uncommon surgical condition. The case highlighted the importance of considering this diagnosis when they encounter a patient with unexplained lower urinary symptoms. Laparoscopic repair is a feasible and safe option if the surgical team was experienced with this approach.

## Introduction

A hernia is an abnormal protrusion of a viscus or part of the viscus through the body wall from the cavity in which it is normally contained. Inguinal hernia repair is one of the most frequently performed operations worldwide, with more than 20 million operations performed for groin hernia repair every year [1]. The lifetime prevalence of inguinal hernia exceeds 40% in men and 5% in women [2]. The risk factor for an inguinal hernia includes advanced age and male sex. Furthermore, there is a positive family history of inguinal hernia in the first-degree relatives. Interestingly, patients with low body weight have a higher tendency to develop inguinal hernia [3]. The inguinal hernia can be due to a congenital or acquired defect. In a congenital inguinal hernia, there is a persistence of processus vaginalis, while the acquired congenital inguinal hernia is due to weakness in the abdominal wall [1]. Clinically, inguinal hernia often presents with a groin swelling with abdominal discomfort [2]. Here, we present a case of inguinal hernia predominantly with urinary symptoms due to the presence of part of the bladder herniating through the inguinal canal, which is an interesting and uncommon clinical finding of inguinal hernia.

## Case presentation

A 39-year-old man presented to our urologic clinic with a complaint of urinary frequency for the last two months. He needed to pass urine every three hours. He also reported that this was associated with a strong desire to pass urine that he cannot defer. The patient was having poor quality of sleep as he needed to awake multiple times every night to pass urine. After urination, he had the feeling of incomplete bladder emptying. He also noted swelling in his right groin. However, he reported that he did not experience any painful urination. There was no history of hesitancy, intermittency, or weak stream. Furthermore, the patient did not experience any penile discharges. The patient visited multiple clinics previously for his complaints and was given symptomatic treatment with oxybutynin, which resulted in minimal improvement in his condition.

The patient was otherwise healthy with no significant previous medical or surgical history. He was not taking any medications and had no known allergies. He was a non-smoker and never consumed alcohol. He worked as an accountant. He had sexual activity with one partner for the last 10 years. The family history was significant for cystic fibrosis. On examination, the patient appeared well and the vital signs were within the normal range. Abdominal examination showed a right groin swelling with associated visible and palpable cough impulse in keeping with inguinal hernia. There was no abdominal guarding or rigidity, and the abdomen was non-tender. Examination of the genitalia was unremarkable. No abnormal findings were noted in the examination of other systems.

Routine laboratory markers did not show any abnormalities (Table 1). The patient had normal leukocytes count with normal values of inflammatory markers. Urinalysis findings showed no leukocytes and had negative results for leukocyte esterase and nitrites. Furthermore, the urine culture had no significant bacterial growth. To further characterize the inguinal swelling, the patient was referred to undergo an abdominal computed tomography (CT) scan. The scan confirmed the presence of a right-sided inguinal hernia. Part of the urinary bladder was herniating into the right inguinal canal. These findings were consistent with inguinal hernia containing part of the urinary bladder (Figure 1).

**Table 1:** Summary of the results of laboratory findings

Laboratory Investigation	Result	Reference Range
Hemoglobin	15.2 g/dL	13.0–18.0
White blood cell	9,200/mL	4.0–11.0
Platelet	375,000/mL	140–450
Erythrocyte sedimentation rate	5 mm/hr.	0–20
C-reactive protein	7.4 mg/dL	0.3–10.0
Total bilirubin	0.9 mg/dL	0.2–1.2
Albumin	4.7 g/dL	3.4–5.0
Alkaline phosphatase	49 U/L	46–116
Gamma-glutamyltransferase	21 U/L	15–85
Alanine transferase	17 U/L	14–63
Aspartate transferase	22 U/L	15–37
Blood urea nitrogen	9 mg/dL	7–18
Creatinine	0.8 mg/dL	0.7–1.3
Sodium	136 mEq/L	136–145
Potassium	4.2 mEq/L	3.5–5.1
Chloride	97 mEq/L	98–107

**Figure 1:** Axial CT images demonstrating right-sided inguinal hernia that contained part of the bladder (arrow). CT, computed tomography

In view of these findings, the patient was referred to the urology team for further management. The decision to undergo surgical repair was taken. The patient underwent a laparoscopic surgery in which the herniated bladder was reduced and the defect was closed with a synthetic mesh. The patient recovered with no complications. Postoperatively, the patient reported significant improvement in his symptoms. He had a close follow-up for six months, and he had no new complaints.

## Discussion

We reported a case of a urinary bladder hernia through the inguinal canal, a rare form of groin hernia. Herniation of the urinary bladder is an uncommon condition and occurs in less than 5% of all inguinal hernias [4]. The first described case of inguinal bladder hernia was reported by Levine in 1951 [5]. A bladder hernia is considered a direct inguinal hernia as it results from an acquired defect in the abdominal wall musculature. It is usually asymptomatic and detected incidentally on imaging studies performed for different indications [4]. However, in our patient, the clinical manifestation was similar to that of an overactive bladder or acute cystitis.

Bladder hernia may get complicated by urinary tract infection, urinary tract obstruction, bladder wall infarction, epididymitis, and malignancy [5]. It is crucial to note that up to 10% of patients with bladder inguinal hernia are diagnosed to have bladder malignancies [4]. In the present case, no such complications were noted and the patient was treated promptly once the diagnosis was made.

Several investigation modalities can be helpful in providing clues for the diagnosis of bladder hernia. Such investigations include ultrasound examination, cystography, CT, and magnetic resonance imaging (MRI) [5,6]. It is interesting to note that less than 10% of patients with bladder hernias are diagnosed preoperatively [4]. The majority of patients with bladder hernias are diagnosed intraoperatively [6]. In the present case, the diagnosis was reached preoperatively as the patient underwent a CT scan as an investigation for his urinary symptoms and groin swelling.

As with all inguinal hernias, bladder inguinal hernia must be repaired surgically once the diagnosis is made to prevent the occurrence of complications [4]. Hernia repair includes reduction of the herniated organ with the closure of the defect either primarily or by using a synthetic mesh material [6]. Partial resection of the bladder might be required in case of bladder infarction [5]. In the present case, the bladder was not displaying any evidence of ischemia, and no resection was performed. The surgical repair can be performed by open laparotomy or laparoscopic repair [5,6]. We used the laparoscopic approach as the surgical team was experienced and confident with this technique and because of its several benefits on patients, including decreased hospital stay.

## Conclusions

Herniation of the bladder through the inguinal canal is an uncommon surgical condition. The case highlighted the importance of considering this diagnosis when they encounter a patient with unexplained lower urinary symptoms. The diagnosis can be reached by cross-sectional imaging modalities. Surgical repair should be performed promptly to avoid the occurrence of complications. Laparoscopic repair is a feasible and safe option if the surgical team was experienced with this approach.
